The article "Role of Parental Smoking in Severe Bronchiolitis: A Hospital Based Case-Control Study" was published in 2017. Journal: Int J Pediatr.

# Role of Parental Smoking in Severe Bronchiolitis: A Hospital Based Case-Control Study

**DOI:** 10.1155/2017/9476367

**Published:** 2017-03-05

**Authors:** Rubina Farzana, Mujibul Hoque, Mohammad Shah Kamal, Md. Moseh Uddin Choudhury

**Affiliations:** ^1^Leprosy Hospital, Sylhet, Bangladesh; ^2^Department of Paediatrics, Sylhet MAG Osmani Medical College, Bangladesh; ^3^Upazila Health Complex, Gowainghat, Sylhet, Bangladesh

## Abstract

*Objective.* Bronchiolitis is one of the commonest causes of hospitalization of infants and young children in Bangladesh. About 21% of under 5 children attending different hospitals of Bangladesh have bronchiolitis. Fifty percent (50%) men and three percent (3%) women of Bangladesh are smokers. Parental smoking is an important risk factor for both susceptibility and severity of bronchiolitis. The aim of this study was to find out the role of parental smoking in severe bronchiolitis.* Design.* Case-control study.* Place and Duration of Study*. The study was conducted in the Department of Paediatrics, Sylhet MAG Osmani Medical College Hospital, Bangladesh, from July 2013 to December 2015.* Patients and Methods*. Sixty-four patients admitted into the ward with severe bronchiolitis were enrolled as cases and sixty-four suitably matched apparently healthy children attending EPI centre and outpatient department presenting with nonrespiratory illness were enrolled as controls. Sample size was calculated using Guilford and Frucher formula. The technique was systematic random sampling. Every second case satisfying the inclusion and exclusion criteria was enrolled in the study.* Results.* The mean age of the patients was 7.53 (SD ± 4.75) months. Forty (62.5%) patients were male and twenty four (37.5%) patients were female. Male-to-female ratio was 1.7 : 1. Most of the cases (60.95%) came from low socioeconomic background. More than half of the cases (53.13%) were not exclusively breastfed babies. Mean length of hospital stay was 6.41 (SD ± 2.82) days. Thirty eight (59%) cases and twenty six (34%) controls were exposed to parental smoking. Result was highly significant (*p* = 0.005). Odds ratio was 2.8 (95% CI from 1.36 to 5.72).* Conclusion.* Exposure to parental smoking causes a statistically significant (*p* = 0.005, odds ratio = 2.8) increase in the risk of developing severe bronchiolitis in the first year of life.

## 1. Introduction

Bronchiolitis is an inflammatory disease of the smallest airways (bronchioles) and is the leading cause of respiratory distress of small children [1]. It is a clinical diagnosis, characterized by cough and respiratory distress associated with wheeze, preceded by runny nose with or without fever in young children below 2 years of age particularly between 2 and 6 months of age [1]. It is predominantly a viral disease. Respiratory Syncytial Virus (RSV) is responsible for more than 50% cases. Other agents include parainfluenza virus, adenovirus, rhinovirus, and mycoplasma [2]. There is no evidence of bacterial cause for bronchiolitis and bronchiolitis is rarely followed by bacterial superinfection [2]. Based on severity of clinical features, bronchiolitis is classified into mild, moderate, and severe [1]. Severe bronchiolitis is characterized by being unable to drink or take feed, severe respiratory distress (chest indrawing, nasal flaring, grunting, and cyanosis), and severe hypoxemia (restlessness, inconsolable cry, and SO_2_ <95%) [1].

About 21% of under 5 children attending different hospitals of Bangladesh have bronchiolitis [3]. Worldwide, 150 million new cases occur annually; 11–20 million (7–13%) of these are severe enough to require hospital admission. 95% of all cases occur in developing countries [4].

Risk factors implicated in the development of severe bronchiolitis include young age, male sex, parental smoking, low socioeconomic background, using of wood burning stoves, and nonbreastfeeding child [1, 5, 6]. Environmental tobacco smoke (ETS) is an important and established risk factor for both susceptibility and severity of bronchiolitis [7].

Currently, there are 1.3 billion smokers in the world [8]. In developed countries, about 35% of men and 22% of women are daily smokers. In developing countries, about 50% of men and 9% of women are daily smokers [8]. In Bangladesh, smoking prevalence is 50% among men and 3% among women [8]. Passive smoking in the family is a major influence in the risk of lower respiratory infections in infants especially on bronchiolitis [9]. Exposure to environmental tobacco smoke had significant association with severe bronchiolitis and prolonged hospitalization [10]. From different studies and observations, it is seen that parental smoking has significant effects in the incidence and severity of acute bronchiolitis. But very few studies are available in our country in this regard. The present study was designed to determine the role of parental smoking in the development of severe bronchiolitis.

## 2. Materials and Methods

### 2.1. Place and Duration of Study

The study was conducted in the Department of Paediatrics, Sylhet MAG Osmani Medical College Hospital, Bangladesh, from July 2013 to December 2015.

### 2.2. Design

It is a case-control study.

### 2.3. Objective

Its objective is to determine the role of parental smoking in the development of severe bronchiolitis.

### 2.4. Diagnosis

After taking a detailed history, clinical examinations were done and severity was assessed according to classification criteria. Chest radiograph was done for the evidence of air trapping in both lungs (hypertranslucency, increased interstitial markings, and hyperinflation). Complete blood counts were done in all the patients. Viral testing (polymerase chain reaction, rapid immunofluorescence, or viral culture) was not done. To differentiate bronchiolitis from pneumonia and asthma, we considered clinical features, white blood cell and differential counts, chest radiograph, and response to bronchodilator.

### 2.5. Treatments

All patients were treated by humidified oxygen with high flow nasal cannula, parenteral fluids, and nebulized salbutamol with or without intravenous corticosteroids. No antibiotics were used.

### 2.6. Sample and Sampling Technique

Sixty-four patients admitted into the ward with severe bronchiolitis were enrolled as cases and sixty-four suitably matched apparently healthy children attending EPI (Extended Programme on Immunization) center and outpatient department presenting with nonrespiratory illness were enrolled as controls. Sample size was calculated using Guilford and Frucher formula. The technique was systematic random sampling. Every second case satisfying the inclusion and exclusion criteria was enrolled in the study.

### 2.7. Demographic Variables

For describing socioeconomic status, we arbitrarily described low (monthly household income <10000 taka), lower-middle (10000–20000 taka), and middle (>20000 taka). The age group was subdivided into three groups: 2–6, 7–12, and 13–24 months.

### 2.8. Data Collection and Analysis

Data were collected in a predesigned case record form. Data were processed and analyzed with the help of statistical package for social sciences [SPSS version 20].

## 3. Results

Sixty-four cases and sixty-four controls were enrolled for this study. The age of the patients ranged from 2 to 24 months with the mean age of 7. 53 (±4.75) months. Most frequent age group was 2 to 6 months (50%) followed by 7–12 months (39%) and 13–24 months (11%). Forty (62.5%) cases were male and 24 (37.5%) cases were female. Male-female ratio was 1.7 : 1. Most of the cases (60.95%) came from low socioeconomic background. More than half of the cases (53.13%) were not exclusively breastfed babies. Minimum length of hospital stay was 3 days and maximum was 10 days; mean hospital stay was 6.41 (±2.82) days. Baseline characteristics between cases and controls did not vary significantly regarding mean age (*p* = 0.452), sex (*p* = 0.370), socioeconomic status (*p* = 0.474), breastfeeding (*p* = 0.859), and use of wood burning stoves (*p* = 0.474) (Table 1).

Among 64 cases, 38 had history of exposure to parental smoking. All exposed cases (38) had history of only paternal smoking and there was no history of maternal smoking or both. Among 64 controls, 22 had history of exposure to parental smoking. The value was highly significant: *p* value = 0.005, odds ratio 2.8 (95% CI from 1.36 to 5.72). So parental smoking carried 2.8 times risk of developing severe bronchiolitis (Table 2).

## 4. Discussion

The age of the patients ranged from 2 to 24 months: most frequent age group was 2–6 months (50%) with the mean age of 7. 53 (±4.75) months. This finding was quite consistent with a study done at the same institute where the mean age of the patients was 5.5 (±3.83) months [11]. Rida [12] found age group 1–6 months as the most frequent (60%) affected group in bronchiolitis. Kabir et al. [6] showed most of the children within 2–12 months (71.5%). Bradley et al. found age as a significant factor in severity of infection; the younger the infant, the more severe the infection [13].

Sex distribution of the patients (male : female; 1.7 : 1) was almost similar to the study of Bashar et al. [11] who found male to female ratio 1.8 : 1. Kabir et al. [6] showed male: female ratio 2.7 : 1. Denicola [14] found males 1.6 times more likely to be hospitalized with bronchiolitis than females, male to female ratio was 1.5 : 1, and death was 1.5 times more likely in males. Semple et al. [15] found male sex significantly associated with severity of the disease. In a Canadian study, male sex was regarded as a strong and independent risk factor for Respiratory Syncytial Virus (RSV) related hospitalization [16]. The reason seems to be of anatomical nature that boys have shorter and narrower airways and are more likely to develop bronchial obstruction in case of RSV infection [17].

In the present study, mean hospital stay was 6.41 (±2.82) days. Kabir et al. [6] found mean length of hospital stay 4.14 (±1.79) days. Bradley et al. [13] found mean hospital stay 2.5 (±2.5) days. Carroll et al. [5] found median length of hospital stay 3 days and infants with maternal smoking had higher risk of having hospitalization >3 days (hazard ratio: 1.38; 95% CI: 1.12–1.71). The prolonged duration of hospital stay found in the current study may be due to peripheral situation of the study institute where both consultant physician and parents of the patients wanted to be more ensured about recovery of the disease.

The present study found exposure to parental smoking in 38 (59%) cases and 26 (41%) controls (*p* = 0.005, odds ratio 2.8). Jones et al. [9] found in their meta-analysis that smoking by either parent or other household members increased the risk of bronchiolitis by an odds ratio of 2.51 (95% CI 1.96–3.21). Chatzimichael et al. [10] found that exposure to environmental tobacco smoke (ETS) carried 2.2 times risk of having severe bronchiolitis (odds ratio = 2.2, 95% CI 1.1–3.6). Semple et al. [15] found the infants from tobacco smoking households at increased risk of severe bronchiolitis needing supplemental oxygen (*p* < 0.001) and mechanical ventilation (*p* < 0.001). Sritippayawan et al. [18] showed environmental tobacco smoke was associated with increased risk of desaturation of the patients (*p* = 0.01). Rida [12] found exposure to passive smoking 2.3 times increased the risk of developing bronchiolitis.

In the present study, all exposed cases of severe bronchiolitis (38 out of 64) had history of only paternal smoking and there was no history of maternal smoking or both. Jones et al. [9] found odds ratio 1.22 (95% CI 1.10 to 1.35) for paternal smoking and 1.62 (95% CI 1.38 to 1.89) for both parental smoking. Strachan and Cook [19] described a causal relationship between parental smoking and acute lower respiratory illness where odds ratios were 1.57 (95% CI 1.42 to 1.74) for smoking by either parent and 1.72 (95% CI 1.55 to 1.91) for maternal smoking. Schvartsman et al. [20] found that children were more affected by maternal smoking (*p* = 0.00016) than paternal one (*p* = 0.015). Jurado et al. [21] described a greater influence of exposure to maternal smoking than paternal smoking in the development of respiratory symptoms in young children.

Limitation of this study was not to estimate urinary “cotinine” level. Cotinine, a major metabolite of nicotine, has been used as a biological marker of smoke absorption to strengthen the evidence of exposure to tobacco smoke

## 5. Conclusion

Exposure to parental smoking, particularly paternal smoking, causes a statistically significant (*p* = 0.005, odds ratio = 2.8) increase in the risk of developing severe bronchiolitis in the first year of life. Protecting young children from parental smoking should be the important approach to prevent the morbidity and mortality caused by severe bronchiolitis.

## Figures and Tables

**Table 1:** Baseline characteristics of the cases and controls (*n* = 64).

Characteristics	Cases	Controls	*p* value
(1) Total number	64	64	
(2) Age in months			0.452^*∗*^
Mean (±SD)	7.53 (±4.75)	8.78 (±5.64)	
(3) Sex			0.370^†^
Male	40 (62.5%)	35 (54.69%)	
Female	24 (37.5%)	29 (45.31%)	
(4) Socioeconomic status			0.474^†^
Low	39 (60.94%)	35 (54.69%)	
Lower-middle	25 (39.06%)	29 (45.31%)	
(5) Breast feeding			0.859^†^
Exclusively breastfed	30 (46.88%)	29 (45.31%)	
Not exclusively breastfed	34 (53.13%)	35 (54.69%)	
(6) Wood-burning stoves users			0.474^†^
Yes	39 (60.94%)	35(54.69%)	
No	25 (39.06%)	29 (45.31%)	

^*∗*^Unpaired “*t*” test was employed to analyze the data.

^†^Chi-Square (*χ*^2^) test was employed to analyze the data.

**Table 2:** Exposure to parental smoking.

Parental smoking	Cases	Controls	*P* value	Odds ratio
Yes	38 (59%)	22 (34%)	0.005	2.8
No	26 (41%)	42 (66%)		
